# MicroRNA let-7c Inhibits Cell Proliferation and Induces Cell Cycle Arrest by Targeting CDC25A in Human Hepatocellular Carcinoma

**DOI:** 10.1371/journal.pone.0124266

**Published:** 2015-04-24

**Authors:** Xiuming Zhu, Lingjiao Wu, Jian Yao, Han Jiang, Qiangfeng Wang, Zhijian Yang, Fusheng Wu

**Affiliations:** 1 Department of Surgical Oncology, the First Affiliated Hospital, College of Medicine, Zhejiang University, Hangzhou, China; 2 Department of Oncology, Zhejiang Provincial People's Hospital, Hangzhou, China; 3 State key Laboratory for Diagnosis and Treatment of Infectious Diseases, the First Affiliated Hospital, College of Medicine, Zhejiang University, Hangzhou, China; 4 Origin Biosciences Inc, Nanjing, China; Harvard Medical School, UNITED STATES

## Abstract

Down-regulation of the microRNA let-7c plays an important role in the pathogenesis of human hepatocellular carcinoma (HCC). The aim of the present study was to determine whether the cell cycle regulator CDC25A is involved in the antitumor effect of let-7c in HCC. The expression levels of let-7c in HCC cell lines were examined by quantitative real-time PCR, and a let-7c agomir was transfected into HCC cells to overexpress let-7c. The effects of let-7c on HCC proliferation, apoptosis and cell cycle were analyzed. The in vivo tumor-inhibitory efficacy of let-7c was evaluated in a xenograft mouse model of HCC. Luciferase reporter assays and western blotting were conducted to identify the targets of let-7c and to determine the effects of let-7c on CDC25A, CyclinD1, CDK6, pRb and E2F2 expression. The results showed that the expression levels of let-7c were significantly decreased in HCC cell lines. Overexpression of let-7c repressed cell growth, induced cell apoptosis, led to G1 cell cycle arrest in vitro, and suppressed tumor growth in a HepG2 xenograft model in vivo. The luciferase reporter assay showed that CDC25A was a direct target of let-7c, and that let-7c inhibited the expression of CDC25A protein by directly targeting its 3ʹ UTR. Restoration of CDC25A induced a let-7c-mediated G1-to-S phase transition. Western blot analysis demonstrated that overexpression of let-7c decreased CyclinD1, CDK6, pRb and E2F2 protein levels. In conclusion, this study indicates that let-7c suppresses HCC progression, possibly by directly targeting the cell cycle regulator CDC25A and indirectly affecting its downstream target molecules. Let-7c may therefore be an effective therapeutic target for HCC.

## Introduction

MicroRNAs (miRNAs) are a class of highly conserved, non-protein-encoding short RNA molecules that repress protein expression through base pairing with the 3′ untranslated region (3′-UTR) of target mRNA [1]. Many reports have shown that miRNAs participate in diverse biological processes [2–4], including the initiation, development and progression of human cancers [5–6]. was previous t Human hepatocellular carcinoma (HCC) is one of the most common malignancies worldwide and is the third most common cause of cancer mortality because of its typically late diagnosis and lack of effective therapies [7]. Similar to other cancers, the development of HCC is a multistep process involving changes of genes and epigenetic alterations. Alteration of miRNA expression is observed in HCC cells and tissues [8–11]. Some miRNAs, such as miR-22, miR-21 and miR-30d, have been shown to play important roles in regulating HCC growth, apoptosis, migration and invasion [12–14]. In humans, 12 genomic loci encode the let-7 family members (let-7a-1, -2, and -3; let-7b; let-7c; let-7d; let-7e; let-7f-1 and -2; let-7g; let-7i and miR-98) [15]. Let-7 is a heterochronic switch gene and regulates developmental timing in Caenorhabditis elegans [16]. In human tumors, let-7 miRNAs are widely viewed as tumor suppressors. Let-7 family members have been found to be down-regulated in lung cancer [17], breast cancer [18], acute lymphoblastic leukemia [19], prostate cancer [20] and HCC [21]. Johnson et al. explored the mechanistic role of let-7 in human lung cancer cells and found that overexpression of let-7 inhibited lung cancer cell proliferation by negatively regulating the expression of RAS [22] and altered cell cycle progression by repressing multiple genes involved in the cell cycle, including CDK6 and cell division cycle 25A (CDC25A) [23]. It has also been reported that let-7c can induce apoptosis and inhibit proliferation of HCC cells in vitro [24]. Our previous study demonstrated that the level of let-7c miRNA was significantly lower in HCC tissues than that in corresponding normal adjacent tumor tissues and that down-regulation of let-7c was correlated with poor tissue differentiation in HCC [25]. These data suggest that let-7c may act as a tumor suppressor in HCC. In this study, we investigated the effects of let-7c on HCC proliferation, apoptosis and the cell cycle in vitro, and on HepG2 xenograft growth in vivo. Furthermore, we determined whether the anti-tumor effect of let-7c is mediated through CDC25A.

## Materials and Methods

### Cell culture

HepG2(no.HB-8065), Hep3B(no.HB-8064) human HCC cells, A549(no.CCL-185) lung cancer cell and HEL 299 (no.CCL-137)human embryonic lung cell were obtained from ATCC. Human HCC cell SMMC-7721,Huh-7 and human immortalized liver cell lines L-02 were obtained from Shanghai Institutes for Biological Sciences of Chinese Academy of Sciences. MHCC97-H and MHCC97-L human HCC cells were obtained from Fudan University (Shanghai, China). The highly metastatic variant, MHCC97-H and the low metastatic potential variant, MHCC97-L are isolated from the parent same cell line. The pulmonary metastatic rates of MHCC97-H and MHCC97-L cell lines are 100% and 40% respectively [26]. HepG2, Hep3B, Huh-7, MHCC97-H, MHCC97-L, A549 and HEL 299 cell lines were cultured with Dulbecco’s modified Eagle Medium. SMMC-7721 and L-02 cell lines were cultured with RPMI 1640. Both media were supplemented with 10%fetal bovine serum and penicillin/streptomycin (GIBCO, Grand Island, NY, USA). All cell lines were incubated at 37°C in a humidified chamber supplemented with 5%CO_2_.

### RNA extraction and quantitative real-time PCR

Total RNA was extracted from HCC cell lines using the mirVana miRNA isolation kit (Ambion, Austin, TX, USA) according to the manufacturer’s instructions. Let-7c expression was measured by using the TaqMan MicroRNA Assay with specific primers for hsa-let-7c (Applied Biosystems, Foster City, CA, USA). U6 snRNA was used for normalization of the relative abundance of let-7c. CDC25A mRNA expression was detected using SYBR Green (Perfect Real Time) (TaKaRa, Otsu, Japan). Glyceraldehyde-3-phosphate dehydrogenase (GAPDH) was used to normalize the CDC25A mRNA expression level. Primers for CDC25A mRNA were as follows: 5′-CTACCTCCCACACTCCCAAG-3′ (forward) and 5′-ACTTCTCTACTCCCCTCCGT-3′ (reverse).

Primers for GAPDH were as follows: 5′-GCTGAGAACGGGAAGCTTGT-3′ (forward) and 5′-GCCAGGGGTGCTAAGCAG-3′ (reverse). Quantitative real-time PCR was performed on an Applied Biosystems 7500 real-time PCR system (Applied Biosystems). Data analyses were performed by using the 2^−ΔΔCt^ method.

### Let-7c agomir and lentiviral vector

Agomirs are a novel class of chemically engineered oligonucleotides. The Let-7 agomir in the present study was cholesterol-conjugated, meaning that the let-7c sequence is cholesterylated, and its effect in cells or tissues is similar to that induced by the overexpression of endogenous let-7c. Cholesterol-conjugated let-7c has higher stability in tissues than a let-7c mimic.

A chemically modified let-7c agomir (5′-UGAGGUAGUAGGGUUGUAUGGUU-3′), a let-7c negative control (5′-CAGUACUUUUGUGUAGUACAA-3′), a let-7c inhibitor (5′-AACCAUACAACCUACUACCUCA-3′) and an inhibitor control (5′-CACCGUUUGUAGCAACUUGUGG-3′) were synthesized by Ribobio (Guangzhou, China). For construction of the let-7c and CDC25A lentiviral vectors, the pre-let-7c sequence or CDC25A gene was amplified and cloned into pLenO-RFP (System Biosciences, Shanghai, China). Virus particles were harvested 48 h following pLenO-RFP–let-7c co-transfection with the packaging plasmids into 293T cells using Lipofectamine 2000 reagent (Invitrogen).

### Cell proliferation assay

The Cell Counting Kit-8 assay (CCK-8, Dojindo, Kumamoto, Japan) was performed to measure the effect of let-7c on cellular proliferation. HepG2, SMMC-7721 or Huh-7 cells were seeded into each well of 96-well plates and incubated overnight, and then transfected with the let-7c agomir at a final concentration of 30 or 50 nM, the negative control or let-7c inhibitor via Lipofectamine 2000 in Opti-MEM (Invitrogen, Carlsbad, CA, USA). Expression of let-7c was detected by using real-time PCR 48 h post transfection. The CCK-8 assay was performed at 24, 48 and 72 h post transfection; 10 μl of the cell proliferation reagent WST-8 was added to each well at the end of the transfection and incubated for 2 h at 37°C. The number of viable cells was determined by reading the optical density at 450 nm.

### Cell apoptosis and cell cycle assays

At 72 h after HepG2, SMMC-7721 or Huh-7 cells were transfected with the let-7c agomir at a final concentration of 30 or 50 nM, the negative control or let-7c inhibitor via Lipofectamine 2000 in Opti-MEM, cell apoptosis was detected by using the Annexin V-PE apoptosis detection kit (BD, USA) according to the manufacturer's protocol. The stained cells were analyzed through fluorescence activated cell sorting (FACS) using BD LSR II flow cytometry (BD Biosciences, San Diego, CA, USA). Apoptosis was determined by calculating the percentage of apoptotic cells relative to the total number of cells. The transfected cells were collected and stained with propidium iodide (PI) for cell cycle analysis with FACS.

### In vivo assay

Animal experiments were performed in strict accordance with the recommendations of the Guide for the Care and Use of Laboratory Animals of the National Institutes of Health. The protocol was approved by the Ethics Committee of the First Affiliated Hospital, College of Medicine, Zhejiang University (Permit Number: 2014–028). All surgeries were performed under sodium pentobarbital anesthesia, and all efforts were made to minimize suffering.

HepG2 cells (2×10^5^) were suspended in 100 μl of PBS and then injected into the flanks of nude mice (BALB/C nu/nu, Kelihua Laboratory Animal Center, Beijing, China) at 5 to 6 weeks of age. In particular, the HCC xenograft model was established after 28 days by injecting the HepG2 cells to form subcutaneous tumors in the nude mice. The mean tumor size was approximately 110 mm^3^. Sixteen tumor-bearing mice were divided at random into a let-7c agomir group and a negative control group, with each group containing 8 mice. Then, 5 nmol of the let-7c agomir or the negative control was injected into each subcutaneous tumor every 3 days. From seventh day after the injection, measurements of tumor size were taken every 7 days for 5 weeks.

To further confirm the anti-tumor effect of let-7c, HepG2 cells were plated to 30–50% confluence and infected with the lentivirus pLenO-RFP-Let-7c or a negative control (pLenO-RFP) using Lipofectamine 2000 in Opti-MEM according to the manufacturer’s instructions; 2×10^5^ infected HepG2 cells were then injected into the flank of a nude mouse. Twenty tumor-bearing mice were divided at random into a Lv-let-7c group (treated with lentivirus pLenO-RFP-let-7c) and a negative control group (treated with pLenO-RFP), with each group containing 10 mice. Tumor-bearing mice were monitored by real-time whole-body fluorescence imaging for tumor growth. Tumor volume was calculated using the formula (L x W^2^) x ½, where W and L represent the perpendicular minor dimension and major dimension, respectively. A fluorescence stereo microscope (MZ650; Nanjing Optic Instrument Inc. China) equipped with D510 long-pass and HQ600/50 band-pass emission filters (Chroma Technology, Brattleboro, VT) and a cooled color charge-coupled device camera (Qimaging, BC, Canada) were used in this experiment. Selective excitation of RFP was achieved through an illuminator equipped with HQ540/40 excitation band-pass filters (Chroma Technology, Brattleboro, VT). Images were processed and analyzed using IMAGE PRO PLUS 6.0 software (Media Cybernetics, Silver Spring, MD).

### Luciferase reporter assay

Putative let-7c targets were identified using the online predictive algorithms TargetScan (http://www.targetscan.org), PicTar (http://pictar.mdc-berlin.de/) and miRanda (http://microrna.sanger.ac.uk) integrated with the miRGen Target program (http://www.diana.pcbi.upenn.edu/miRGen.html). CDC25A was selected as a potential target of let-7c. The let-7c binding sites at the CDC25A 3′-UTR were amplified by PCR from HEK-293 cell genomic DNA and cloned into the XhoI and NotI sites downstream of the luciferase reporter gene in the pmiR-RB-Report vector (pmiR-CDC25A-3′-UTR-wt). Three mutant constructs were generated using a KOD-Plus-mutagenesis kit (TOYOBO, Osaka, Japan). All constructs were verified by DNA sequencing. HepG2 cells were co-transfected with pmiR-CDC25A-3′-UTR-wt or pmiR-CDC25A-3′-UTR–mut reporters along with either the let-7c agomir or negative control in 96-well plates by using Lipofectamine 2000. Luciferase activity was measured by using the dual luciferase assay system (Promega, Heidelberg, Germany) 48 h post transfection. Renilla luciferase was used as an internal control; the firefly luciferase activity of each sample was normalized to the activity of Renilla luciferase. The experiment was performed independently in triplicate.

### Western blot assay

HepG2,SMMC-7721 or Huh-7 cells transfected with the let-7c agomir or inhibitor at a final concentration of 50 nM were harvested 72 h post transfection. HepG2, SMMC-7721 or Huh-7 cells were infection/transfection with lenti-CDC25A, lenti-control, CDC25A-siRNA or negative control-siRNA. Total protein from the infected/transfected HCC cells was extracted by using standard protocols. The target protein levels were determined using primary antibodies against CDC25A, cyclin-dependent kinase 6 (CDK6), CyclinD1, pRb, Rb, E2F2 and β-actin (Abcam, Cambridge, UK). The values for these proteins were normalized to the corresponding values for ß-actin or actin. Band signals were acquired in the linear range of the scanner and analyzed using QUANTITY ONE software (Bio-Rad, Hercules, CA, USA).

### Immunohistochemistry (IHC)

Fresh mouse tumor tissues were collected, formalin-fixed and paraffin-embedded. The tissues were cut into 5-μm sections, placed in dimethylbenzene, rehydrated through graded ethanol solutions, exposed to 0.3%hydrogen peroxide and processed by microwave heating in 10 mM citrate buffer for antigen retrieval. Sections were incubated at 4°C overnight with anti-CDC25A mouse mAb (Abcam, Cambridge, UK). PBS was used rather than the primary antibody as a negative control. Immunostaining was performed using a ChemMate EnVision Detection Kit (DAKO) according to the manufacturer’s instructions. Ten areas were randomly selected and counted at a magnification of 400. CDC25A staining was evaluated semi-quantitatively on the basis of the percentage of positive cells and classified as follows: intensely positive (+++) when positive cells comprised more than 50% of the total cells; moderately positive (++) when positive cells comprised 16–50%; weakly positive (+) when positive cells comprised 10–15%; and negative (-) when positive cells comprised less than 10% [27].

### Statistical analysis

Data were presented as the mean ± SD from at least three independent experiments. Statistical analyses were performed using SPSS16.0 software. Two or multiple group comparisons were performed using Student’s t-test or ANOVA. P<0.05 was regarded as statistically significant and indicated with *.

## Results

### Decreased expression of let-7c in HCC cell lines

Our previous study found that let-7c expression was significantly down-regulated in HCC tumors compared to paired normal adjacent tissues [25]. As shown in Fig 1, expression of let-7c was significantly decreased in the HCC cell lines HepG2, Hep3B, SMMC-7721,Huh-7, MHCC97-H and MHCC97-L compared to the normal liver cell line L-02 (P<0.01). Moreover, the let-7c expression of MHCC97-H cells (high metastatic potential) was lower than that of MHCC97-L cells (low metastatic potential). The expression of let-7c in A549 lung cancer cells was also lower than that in the human embryonic lung cell line HEL 299.

**Fig 1:** Let-7c is down-regulated in various HCC cell lines. Let-7c expression levels in various HCC cell lines (HepG2, Hep3B, SMMC-7721,Huh-7, MHCC97-H, and MHCC97-L), the normal human liver cell line L-02, A549 lung cancer cells and HEL 299 cells (human embryonic lung cell) were determined by quantitative real-time PCR. Each sample was analyzed in triplicate and normalized to U6 expression.

### Over-expression of let-7c inhibits HCC cell proliferation and induces apoptosis, leading to G1 cell cycle arrest in vitro

HepG2 and SMMC-7721 cells were transfected with the let-7c agomir or negative control to investigate the effects of over-expression of let-7c on cell proliferation and the cell cycle. Expression of let-7c was significantly increased in HepG2 and SMMC-7721 cells transfected with the let-7c agomir compared to cells transfected with the negative control (Fig 2A). Tumor cell proliferation was significantly inhibited by overexpression of let-7c via the let-7c agomir at 48 h post transfection (Fig 2B). The inhibition of cell proliferation by let-7c agomir overexpression was concentration-dependent. Furthermore, overexpression of let-7c in HepG2 and SMMC-7721 HCC cells significantly induced tumor cell apoptosis 72 h post transfection (Fig 2D) and inhibited cell cycle progression, leading to G1-phase arrest, compared to the negative control (Fig 2C). In addition, Huh-7 cells were also transfected with the let-7c agomir or negative control, overexpression of let-7c significantly inhibited Huh-7 cells proliferation and induced apoptosis. The results were similar to the one that in HepG2 and SMMC-7721 cells. However, the proliferation of Huh-7 cells increased and the number of apoptotic cells decreased when endogenous let-7c was silenced using the let-7c inhibitor (S1A and S1B Fig).

**Fig 2:** Let-7c inhibits HCC cell proliferation, induces cell apoptosis and induces G1 cell cycle arrest in vitro. (A) HepG2 and SMMC-7721 HCC cells were transfected with the let-7c agomir at a final concentration of 30 or 50 nM. Expression of let-7c was determined using quantitative real-time PCR 48 h post-transfection. (B-D) HepG2 and SMMC-7721 HCC cells were transfected as in (A). At the indicated time points post transfection, the cell growth rate was evaluated using the CCK-8 assay (B). Cells were stained using propidium iodide (PI) and Annexin V 72 h post transfection and analyzed by FACS. Annexin V-positive cells were regarded as apoptotic cells (D) and the cell cycle distribution was calculated (C).

### Let-7c inhibits tumor growth in a xenograft mouse model of HCC

To investigate the anti-tumor effect of let-7c in vivo, an HCC xenograft model was established by injecting HepG2 cells to form subcutaneous tumors in nude mice. Injection of the let-7c agomir significantly inhibited tumor growth compared to the control group (Fig 3A, 3B and 3C). To further confirm the anti-tumor effect of let-7c, HepG2 cells infected with the lentivirus pLenO-RFP-let-7c (Lv-let-7c) or pLenO-RFP (Lv-control; negative control) were implanted into the flanks of nude mice. Tumor growth was measured by real-time whole-body fluorescence imaging to evaluate the effect of let-7c on tumor inhibition. The tumor size was significantly reduced in the group infected with pLenO-RFP-Let-7c compared to the group infected with pLenO-RFP (negative control; Fig 4A and 4D). Tumor weight in the pLenO-RFP-let-7c group was significantly lower than that in the negative control (Fig 4C). Additionally,let-7c expression level in tumor tissues transfected with pLenO-RFP-let-7c was significantly higher than that in tissues transfected with pLenO-RFP (Fig 4B).

**Fig 3:** Let-7c agomir inhibits tumor growth in a xenograft mouse model of HCC in vivo. (A) Photographs of tumor-bearing mice in the fifth week after injection with let-7c agomir (Left) or negative control (Right). (B) From seventh day after the injection, measurements of tumor size were taken every 7 days for 5 weeks. Effects of let-7c agomir on the xenograft mouse model are shown. Data are shown as the mean ± S.D. The statistical difference was analyzed by the two-sample t test. (C) Photographs of tumors that developed in the mouse model of HCC treated with let-7c or the negative control are presented. The two smallest tumors with the let-7c treatment are indicated by red arrows, and the two smallest tumors in the negative control group are indicated by blue arrows.

**Fig 4:** pLenO-RFP-Let-7c inhibits tumor growth in a xenograft mouse model of HCC in vivo. (A) Effects of pLenO-RFP-let-7c (Lv-let-7c) and pLenO-RFP (Lv-control, negative control) in the xenograft mouse model are shown. Data are shown as the mean ± S.D. The statistical difference was analyzed by the two-sample t test. (B) qRT-PCR assays of mature let-7c expression in tissues of the Lv-let-7c and Lv-control group. (C) Weight of tumors of mice in the Lv-let-7c and Lv-control groups. Data are shown as the mean ± S.D. The statistical difference was analyzed by the two-sample t test. (D) Photographs of tumors are presented. The three smallest tumors in the Lv-let-7c group are indicated by blue arrows.

### CDC25A is a direct target of let-7c

To investigate the underlying the molecular mechanism through which let-7c induces a G1 cell cycle arrest, potential targets of let-7c were predicted using the algorithms PicTar, miRanda and TargetScan. Fifty-eight candidate genes were predicted by all three algorithms to be possible targets of let-7c (S2 Fig). Of these fifty-eight candidate genes, CDC25A has been shown to play a critical role in transition through the G1 to S checkpoint (S1 Table). As shown in Fig 5A, the 3′UTR of CDC25A mRNA contained two complementary sites for the seed region of let-7c. Luciferase reporter assay and western blot analysis were performed to determine whether CDC25A is a direct target of let-7c in HCC. Firefly luciferase reporter vectors containing the CDC25A wild-type (pmiR-CDC25A-3′-UTR-wt) or mutant (pmiR- CDC25A-3′-UTR–mut) 3′-UTR were generated and co-transfected into HepG2 cells along with either the let-7c agomir or negative control (Fig 5A). The luciferase activity of the reporter vector containing the CDC25A wild-type 3′-UTR was significantly inhibited by co-transfection with the let-7c agomir compared to the negative control. No inhibitory effect was found for the vector containing a mutated binding site (Fig 5B).

**Fig 5:** Let-7c targets CDC25A in HCC cells. (A) Firefly luciferase reporter vectors containing the CDC25A wild-type (pmiR-CDC25A-3′-UTR-wt) or mutant (pmiR- CDC25A-3′-UTR–mut) 3′-UTR were generated and co-transfected into HepG2 cells along with either the let-7c agomir or negative control to identify CDC25A targets. The 3′UTR of CDC25A mRNA contained two complementary sites for the seed region of let-7c. (b) Wild: wild-type; Mut: mutated. The seed sequence is underlined. (B) Relative luciferase activity was analyzed after the reporter plasmids or control reporter plasmid were co-transfected with let-7c into HEK-293 cells. Representative experiments are shown. (C) Western blot assays of the endogenous CDC25A protein level in HepG2 cells transfected with the let-7c agomir, negative control or let-7c inhibitor. (D) Real-time PCR assay of CDC25A mRNA expression in HepG2 cells transfected with the let-7c agomir or negative control.

CDC25A protein expression in HepG2 cells was significantly decreased by transfection with the let-7c agomir and increased by transfection with the let-7c inhibitor compared to the corresponding controls (Fig 5C). However, the expression of CDC25A mRNA was not significantly influenced by the let-7c agomir (Fig 5D), suggesting that CDC25A expression is inhibited by let-7c mainly at the post-transcriptional level.

### Restoration of CDC25A induces let-7c-mediated G1-to-S phase transition in HCC cells

To explore the role of CDC25A in let-7c-mediated suppression of tumorigenesis, HepG2 cells were infected with a lentiviral construct containing the CDC25A gene or vector alone (Fig 6A). Overexpression of CDC25A induced a G1-to-S phase transition in HepG2 cells (Fig 6D). In addition, knockdown of CDC25A expression by siRNA in HepG2 cells resulted in G1 phase arrest (Fig 6B and 6E) similar to that induced by overexpression of let-7c. However, overexpression or knockdown of CDC25A had only a slight influence on HepG2 cell apoptosis (S3A Fig).

**Fig 6:** CDC25A induces the G1-to-S phase transition in HCC cells. (A,B) Western blotting of CDC25A protein expression in HepG2 cells infected/transfected with lenti-CDC25A, lenti-control, CDC25A-siRNA or negative control-siRNA. (C) Western blot analysis of CDC25A expression in SMMC-7721 cells and SMMC-7721-let-7c stable cells with or without CDC25A* reintroduction. (D,E) Infection/transfection of HepG2 cells with lenti-CDC25A, lenti-control, CDC25A-siRNA or negative control-siRNA was performed to investigate the effects of CDC25A on the HCC cell cycle. Representative images are shown. (F) Cell cycle assays of SMMC-7721 cells or SMMC-7721-let-7c stable cells with or without CDC25A* reintroduction. Restoration of CDC25A significantly induced the G1-to-S phase transition in SMMC-7721 cells. Representative images are shown. *CDC25A was reintroduced without its 3′-UTR to prevent the expression of CDC25A from being inhibited by let-7c.

To further verify that down-regulation of CDC25A is involved in let-7c-mediated suppression of tumorigenesis, we reintroduced CDC25A without its 3′-UTR, to prevent the expression of CDC25A from being inhibited by let-7c. The restoration of CDC25A protein expression in SMMC-7721-let-7c stable cells was confirmed by western blot (Fig 6C), and it significantly induced the G1-to-S phase transition initiated by let-7c in SMMC-7721 cells (Fig 6F). However, the number of apoptotic SMMC-7721 cells did not change significantly following the restoration of CDC25A, perhaps because let-7c regulates other targets such as Bcl-xl that affect apoptosis (S3B Fig).

### Let-7c down-regulates CDC25A, CDK6, CyclinD1, pRb and E2F2 proteins

As CDC25A directly phosphorylates and activates CDKs by removing inhibitory phosphorylation, leading to the differential expression of their downstream target proteins, the expression levels of CDK6, CyclinD1, pRb and E2F2 proteins were assayed. HepG2 and SMMC-7721 cells were transfected with the let-7c agomir, let-7c inhibitor or a negative control. CDK6, CyclinD1, pRb and E2F2 proteins were significantly down-regulated by transfection with the let-7c agomir in HepG2 and SMMC-7721 cells compared to cells transfected with the negative control. Transfection with the let-7c inhibitor increased the expression of CDK6, CyclinD1, pRb and E2F2 proteins (Fig 7A). In mouse xenograft tumors derived from pLenO-RFP-Let-7c-infected HepG2 cells, CDC25A protein expression was decreased (Fig 7B). As shown in Table 1, the tumors infected with pLenO-RFP-Let-7c showed a higher rate of negative CDC25A staining (50%) than the tumors infected with the control vector (20%).

**Fig 7:** Effect of Let-7c on CDC25A, CDK6, CyclinD1, pRb, Rb and E2F2 protein expression in HCC cells. (A) HepG2 and SMMC-7721 cells were transfected with the let-7c agomir, let-7c inhibitor or negative control. Levels of CDC25A, CDK6, CyclinD1, pRb, Rb and E2F2 protein were detected by western blot. The value under each band indicates the relative expression levels of CDC25A, CDK6, CyclinD1, pRb, Rb and E2F2 compared to actin. (B) Immunohistochemistry was performed to determine CDC25A protein expression in HCC xenograft tumor tissues. Images were captured at 40×10 magnification. Positive CDC25A expression was observed as brown particles in the cytoplasm and the nucleus.

**Table 1:** Effect of let-7c on CDC25A protein expression in HCC xenograft tumors.

CDC25A protein expression	Negative(-)	Weak(+)	Moderate(++)	Strong(+++)
**Control**	2/10(20%)	4/10(40%)	3/10(30%)	1/10(10%)
**Let-7c**	5/10(50%)	4/10(40%)	1/10(10%)	0/10(0)

Immunohistochemical analyses show the effect of let-7c on CDC25A protein expression in HCC xenograft tumors infected with lentiviral pLenO-RFP-Let-7c or the pLenO-RFP negative control.

## Discussion

In this study, we found that let-7c expression was decreased in HCC cell lines. Over-expression of let-7c inhibited HCC cell proliferation, induced cell apoptosis and led to G1 phase arrest in vitro, and it suppressed the tumor growth of HCC xenografts in vivo. These results demonstrate that let-7c functions as a tumor suppressor that inhibits HCC tumor growth, mainly by regulating the cell cycle. It is known that cell cycle deregulation is a common feature of human cancer [28], as cancer cells frequently display unscheduled proliferation resulting from disruptions of cell cycle such as G1-phase arrest. Emerging evidence suggests that some miRNAs could directly or indirectly target transcripts that encode proteins involved in cell cycle progression [29]. It has been reported that miR-106b contributes to the inhibition of tumor cell proliferation by regulating the cell cycle checkpoint molecule P21 [30]. Johnson reported that let-7c inhibits lung cell proliferation by regulating multiple genes involved in the cell cycle, including CDK6 and CDC25A [23]. Let-7c has also been reported to induce HCC cell apoptosis and to inhibit the proliferation of Huh7 and HepG2 cell lines in vitro [24]. Over-expression of miR-24 increases the percentage of cells in the G1 phase and inhibits cell proliferation in HepG2 and K562 tumor cells [31]. Gong reported that Let-7c inhibits the proliferation of LM3 HCC cells and expression of cyclin D1, and it increases the proportion of cells in the G1 phase [32]. These results are consistent with our finding that let-7c suppresses cyclin D1/CDK6, leading to G1 phase arrest in HepG2 and SMMC-7721 cells.

CDC25A is one of the most crucial cell cycle regulators; it removes the inhibitory phosphorylation of cyclin-dependent kinases (CDKs) such as CDK2, CDK4 and CDK6 and positively regulates the activity of CDKs that lead to cell cycle progression, including the transition from the G1 to the S phase [33, 34]. Up-regulation of CDC25A protein is commonly observed in various types of cancer, including HCC [35, 36], and is correlated with shorter survival of HCC patients [37]. Our study showed that CDC25A is a direct target of let-7c in HCC; cellular CDC25A expression was decreased at the protein level through transfection with let-7c, which directly bound to the 3′UTR, but not at the mRNA level, indicating that let-7c functions by regulating the protein level of CDC25A mainly at the post-transcriptional level. It has been reported that miRNA-mediated suppression of protein production occurs through a mechanism that operates after the initiation of protein synthesis. Therefore, the reduction of protein production may not be accompanied by corresponding changes in mRNA expression [38, 39].

Activation of CDC25 is considered to be the trigger that activates cyclin-CDK, initiating the next phase of the cell cycle. It has been found that CDK6/cyclin D phosphorylates pRB and related pocket proteins, allowing them to disassociate from E2F. Activated E2F proteins can then transcribe S phase-promoting genes [40]. The deregulation of cell signaling pathways such as Rb-E2F plays an important role in cell proliferation and cell fate determination [41,42]. Alterations in E2F function coincide with a poor prognosis in cancers, emphasizing their importance for the clinical cancer phenotype [43]. The activity of E2F is regulated by some miRNAs, and in turn, miRNAs themselves are targets of proteins in the E2F family [43]. It has been reported that miR-195 blocks the G1/S transition by repressing Rb-E2F signaling through targeting of multiple molecules, including cyclin D1, CDK6, and E2F3 [41]. MiR-17 and miR-20a may block the G1/S transition by repressing Rb-E2F signaling by directly targeting E2F1 molecules in normal diploid human cells [44], and miR-34a induces senescence-like growth arrest through modulation of the E2F pathway in human colon cancer cells [45]. Dong et al. reported that the anti-proliferative mechanism of let-7a is related to the down-regulation of E2F2 and CCND2 in prostate cancer [46]. Our study found that over-expression of let-7c inhibited the activation of CDK6, pRb and E2F2 and that, conversely, inhibition of let-7c enhanced the expression of these proteins, indicating that let-7c suppressed the expression of CDC25A protein and subsequently led to the down-regulation of CDK6, CyclinD1, pRb and E2F2 proteins in human HCC.

## Conclusions

This study demonstrates that let-7c inhibits cell proliferation and induces cell cycle arrest possibly by directly targeting CDC25A and indirectly affecting its downstream target molecules (e.g., CDK6, pRb, and E2F2) in HCC. These results suggest that let-7c is a potential therapeutic target for HCC.

## Supporting Information

S1 Fig Effect of Let-7c on Huh-7 cells proliferation and apoptosis. Huh-7 cells were transfected the let-7c agomir, let-7c inhibitor or negative control. (A)At the indicated time points post transfection, cell growth rate was evaluated using the CCK-8 assay.(B)Cells were stained using propidium iodide (PI) and Annexin V 72 h post-transfection and analyzed by FACS. The Annexin V-positive cells were regarded as apoptotic cells.
(TIF)

S2 Fig Schematic representation of the candidate genes predicted by three prediction algorithms. Each labeled circle represents one prediction algorithm with the number of its predicted genes, and the number listed in the overlapping regions of the circles is the number of targets commonly predicted by different algorithms.
(TIF)

S3 Fig Effect of CDC25A on HCC cell apoptosis. (A)HepG2 cells infected/transfected with lenti-CDC25A or lenti- control and CDC25A-siRNA or negative control-siRNA were used to investigate the effects of CDC25A on HCC cell apoptosis. Representative images are shown. (B)Cell apoptosis assays for SMMC-7721 cells or SMMC-7721-let-7c stable cells with or without CDC25A* reintroduction. Representative images are shown.
(TIF)

S1 Table The name and information are listed for the 58 predicted genes. Potential targets of let-7c were predicted using the algorithms PicTar, miRanda and TargetScan.
(DOC)
